The article "Account of Deep Learning-Based Ultrasonic Image Feature in the Diagnosis of Severe Sepsis Complicated with Acute Kidney Injury" was retracted in 2023. Reasons: signs of a paper mill; suspected computer-generated content; unreliable results or conclusions; concerns about the data.

# Account of Deep Learning-Based Ultrasonic Image Feature in the Diagnosis of Severe Sepsis Complicated with Acute Kidney Injury

**DOI:** 10.1155/2022/8158634

**Published:** 2022-01-31

**Authors:** Yi Lv, Zhijia Huang

**Affiliations:** Department of Critical Care Medicine, The Second Affiliated Hospital, Hengyang Medical University, University of South China, Hengyang, 421001 Hunan, China

## Abstract

This study was aimed at analyzing the diagnostic value of convolutional neural network models on account of deep learning for severe sepsis complicated with acute kidney injury and providing an effective theoretical reference for the clinical use of ultrasonic image diagnoses. 50 patients with severe sepsis complicated with acute kidney injury and 50 healthy volunteers were selected in this study. They all underwent ultrasound scans. Different deep learning convolutional neural network models dense convolutional network (DenseNet121), Google inception net (GoogLeNet), and Microsoft's residual network (ResNet) were used for training and diagnoses. Then, the diagnostic results were compared with professional image physicians' artificial diagnoses. The results showed that accuracy and sensitivity of the three deep learning algorithms were significantly higher than professional image physicians' artificial diagnoses. Besides, the error rates of the three algorithm models for severe sepsis complicated with acute kidney injury were significantly lower than professional physicians' artificial diagnoses. The areas under curves (AUCs) of the three algorithms were significantly higher than AUCs of doctors' diagnosis results. The loss function parameters of DenseNet121 and GoogLeNet were significantly lower than that of ResNet, with the statistically significant difference (*P* < 0.05). There was no significant difference in training time of ResNet, GoogLeNet, and DenseNet121 algorithms under deep learning, as the convergence was reached after 700 times, 700 times, and 650 times, respectively (*P* > 0.05). In conclusion, the value of the three algorithms on account of deep learning in the diagnoses of severe sepsis complicated with acute kidney injury was higher than professional physicians' artificial judgments and had great clinical value for the diagnoses and treatments of the disease.

## 1. Introduction

Now, as sepsis is better understood, it is defined by scholars as a clinical syndrome in which organism's inflammatory response is maladjusted by infection, resulting in severe damage to physiology and organ functions. Sepsis has extremely high morbidity and mortality in intensive care units, and it has become the leading cause of death for critically ill patients [1]. According to some studies, there are more than 30 million new cases of concentrated diseases in the world every year, and more than five million people have been killed by sepsis, which have caused serious pressure and burden on global public health [2–4]. Its pathogeneses and pathological processes are complicated and closely related to inflammation, coagulation dysfunction, and immune disorders [5–7]. Among them, uncontrolled inflammatory response is considered to be one of the pathogeneses of sepsis. Early inflammatory responses released a large amount of proinflammatory cytokines and anti-inflammatory cytokines [8]. However, there is often an imbalance between proinflammatory factors and anti-inflammatory factors in sepsis patients, and the inflammatory reaction is out of control, which accelerates the development of sepsis [9–11]. In addition, inflammation often interacts with coagulation dysfunction and then influences the development of sepsis. The decreased expression of tissue factors cannot initiate the exogenous coagulation pathway, which results in coagulation disorders and accelerates the formation of vascular damage [12–14].

The article "Account of Deep Learning-Based Ultrasonic Image Feature in the Diagnosis of Severe Sepsis Complicated with Acute Kidney Injury" was retracted in 2023. Reasons: signs of a paper mill; suspected computer-generated content; unreliable results or conclusions; concerns about the data.

Acute kidney injury is usually characterized by rapid decline in renal function, which results in acute kidney failure and other organ failure in severe cases. Acute kidney injury can be caused by a variety of factors, which include drug use, ischemia/reperfusion, and infection [15–17]. In recent years, the incidence and mortality of acute kidney injury have been increasing, and the mortality rate of severe acute kidney injury can reach more than 50%. The pathogeneses of acute kidney injury are often related to their pathogenic factors. During organ transplantation, acute blood loss, or toxic shock, ischemia/reperfusion injury has become an important pathogenic mechanism which leads to acute kidney injury [18]. As the most important excretory organ in the human body, drugs are often excreted through the kidney, and their massive use or even abuse is likely to cause drug-induced acute kidney injury [19]. Sepsis complicated with acute kidney injury refers to acute renal parenchymal injury occurring to patients with sepsis, and other factors may cause kidney damage like renal ischemia or nephrotoxic substances are excluded. Acute kidney injury is quite common in people with sepsis, and the incidence increases with the severity of sepsis. Epidemiological data show that the incidence of acute kidney injury is 19%, 23%, and 51% in patients with moderate sepsis, severe sepsis, and septic shock, respectively. In view of the high incidence of sepsis, it can be estimated that the number of acute kidney injury cases induced by sepsis is quite alarming. Compared with other causes, sepsis gives more unstable hemodynamics of acute kidney injury; the proportion of patients who need vasopressors and mechanical ventilation is higher, the disease severity score is higher, and the mortality is also significantly increased ultimately. Delays in early diagnoses and treatments lead to continuous progression of the disease, and continuous hypoperfusion leads to acute tubular necrosis, which eventually develops into irreversible damage, even patients' death [20–22].

The article "Account of Deep Learning-Based Ultrasonic Image Feature in the Diagnosis of Severe Sepsis Complicated with Acute Kidney Injury" was retracted in 2023. Reasons: signs of a paper mill; suspected computer-generated content; unreliable results or conclusions; concerns about the data.

Clinically, early diagnoses are often made by creatinine and urine volume detections according to international guidelines, but it is usually unable to making correct diagnoses in time and completely. With the continuous development of image examination, ultrasound image examination is gradually applied in the clinical diagnoses of sepsis complicated with acute kidney injury. Clinical workers are often unable to sum up quantitative and accurate medical information from ultrasonic images by naked eyes. Medical image analyses and processing technologies solve this dilemma and become important helpers of clinical diagnoses [23–25]. The purpose of further analyses and clarification is to help clinicians diagnose the disease more accurately and quickly and obtain more in-depth information of the disease. Convolutional neural network, a kind of deep neural network, consists of a deeper grid structure which is able to read image data as visual pathological features and find features that human eyes cannot read. This is very important for ultrasonography in the diagnoses of sepsis complicated with acute kidney injury.

This study was intended to analyze the diagnostic value severe sepsis complicated with acute kidney injury under deep learning-based convolutional neural network, to provide a certain reference for the clinical ultrasound image diagnosis.

## 2. Materials and Methods

### 2.1. Study Objects

In this study, 50 patients with severe sepsis complicated with acute kidney injury admitted to hospital from January 10, 2020, to May 10, 2021, were selected as the experimental group. According to the age and gender distribution of these patients, 50 healthy volunteers were also selected as the healthy control group. This study had been approved by ethics committee of hospital, and patients' families had been informed of this study and signed informed consents.

Inclusion criteria were as follows. First, patients were diagnosed as sepsis complicated with acute kidney injury according to the diagnostic criteria. Second, patients had signed informed consent forms. Third, patients did not suffer from other serious organ diseases or hereditary diseases. Fourth, patients were not examined for contraindications.

The article "Account of Deep Learning-Based Ultrasonic Image Feature in the Diagnosis of Severe Sepsis Complicated with Acute Kidney Injury" was retracted in 2023. Reasons: signs of a paper mill; suspected computer-generated content; unreliable results or conclusions; concerns about the data.

The patients met exclusion criteria had severe allergies, other serious underlying diseases, and a history of chronic kidney injury. Moreover, the patients took diuretics for a long time.

There were two requirements in the criterion for suspension and elimination. First, patients could not normally complete ultrasound scans. Second, patients who did not comply with the treatments were followed up for index evaluation.

For healthy control group volunteers, the inclusion criterion was the same as those for patients with sepsis complicated with acute kidney injury (2^nd^-4^th^). The exclusion criterion was the same as those for patients with sepsis complicated with acute kidney injury (2^nd^-4^th^). Patients with acute kidney injury complicated with sepsis were discontinued and excluded.

### 2.2. Ultrasonic Image Examinations

Ultrasound image examinations were performed in 100 patients at the same time. The patients should be examined with empty stomachs, did not drink a lot of water before the examination, and lay on the examination bed in the supine position and the left lateral position. Ultrasound system and convex array 3.5 MHZ probe were applied for renal ultrasound examination. The probe was placed in the posterior axillary line, and the position and angle of the probe were adjusted to get the largest coronal image of the kidney. The probe was rotated in 90° at the coronal section and was moved up and down to adjust the angle of the sound beam, then the cross-sectional image of the kidney was obtained. When the patients were in the prone position, the probe was placed under the ribs of the back for longitudinal scanning. With the probe mark facing towards the head, the sagittal plane of the kidney could be observed.

### 2.3. Convolutional Neural Network Models

The DenseNet121 convolutional neural network structure models completed classification processes through convolution, maximum pooling layers, dense modules, and complete connection layers, respectively. Due to the tight connection between different levels, DenseNet121 model could absorb and use features of each level and overcome problems of gradient disappearance to a certain extent. The specific grid structure model of DenseNet121 was shown in Figure 1.

In the structure model of GoogLeNet convolutional neural network, the number of network layers was significantly increased, but there were few parameters. There was an integrated inception module which could combine pooling layer and convolution layer to achieve fast computing speed and obtain more feature information. Additionally, there were a large number of inception branches. Their structures and characteristics were different, and the final calculation results were more accurate. The inception module of GoogLeNet was shown in Figure 2.

The article "Account of Deep Learning-Based Ultrasonic Image Feature in the Diagnosis of Severe Sepsis Complicated with Acute Kidney Injury" was retracted in 2023. Reasons: signs of a paper mill; suspected computer-generated content; unreliable results or conclusions; concerns about the data.

ResNet was an excellent object detection, image classification, and segmentation model which had been widely used in convolutional neural networks. Residual structures appeared in ResNet model, which made it easier to optimize. In the propagation process of neural network, the propagation gradient gradually disappeared due to the appearance of back propagation. Since the existence of residual structures solved this problem, the gradient information was more easily transmitted in the process of reverse transmission of residual structures, and the network with residual modules would get higher identification accuracy. At the same time, ResNet residual network model adopted a large number of relatively standardized method enzyme training. Its specific structural model was shown in Figure 3.

ResNet improved the number of network layers through residual structures and simplified the learning objects to realize the improvement of training speed and the accuracy of parameters. It was suggested to input the initial value *x*_*i*_ and set the weight to *a*. The bias was represented by *c*, *y*_*i*_ was the branch sum, and its calculation functions were shown in the following equations:

(1) $$\begin{array}{c} F\left(x_{i}\right)=ax_{i}+c, \end{array}$$

(2) $$\begin{array}{c} y_{i}=M\left(F\right)+v\left(x_{i}\right), \end{array}$$

(3) $$\begin{array}{c} x_{i+1}=M\left(y_{i}\right). \end{array}$$

The activation function could avoid gradient dispersion problems and reduce gradient attenuation, which was shown in the following equation:

(4) $$\begin{array}{c} M\left(b\right)=\max\left(0,b\right). \end{array}$$

When *b* > 0, *M*(*b*) = *b*, its derivative was 1. When *b* < 0, *M*(*b*) = 0, its derivative was 0. When *b* = 0, *M* of *b* was equal to 0; its derivative was 0.

The cross entropy was used as the loss function, *o* and *p* were two normal probability distributions. The cross entropy of *o* was represented by *p* in the figure. It was shown in the following equation:

(5) $$\begin{array}{c} M\left(o,p\right)=-\sum o\left(a\right)\log p\left(a\right). \end{array}$$

Cross entropy must satisfy the probability distribution function, which were shown in the following equations:

(6) $$\begin{array}{c} \forall ao\left(X-a\right)\in \left[0,1\right], \end{array}$$

(7) $$\begin{array}{c} \sum o\left(X-a\right)=1. \end{array}$$

### 2.4. Evaluation Criteria

In this study, ultrasonic images of three common indicators on account of deep learning were used to evaluate the diagnostic effect of severe sepsis complicated with acute kidney injury. Three common indicators were accuracy, specificity, and sensitivity. Calculation methods were shown in the following equations:

(8) $$\begin{array}{c} \text{Accuracy}=\frac{A+B}{A+C+B+D}, \end{array}$$

(9) $$\begin{array}{c} \text{Specificity}=\frac{B}{C+B}, \end{array}$$

(10) $$\begin{array}{c} \text{Sensitivity}=\frac{A}{D+A}. \end{array}$$

In addition, the diagnosis error rate of ultrasonic images on account of deep learning was shown in the following equation:

(11) $$\begin{array}{c} M=\frac{C+D}{A+B+C+D}. \end{array}$$

*A* was true positive, indicating that the diagnosis result was positive, which was actually positive. *B* was true negative, meaning that the diagnosis was negative, which was truly negative. *C* was false positive, indicating that the diagnosis was positive, but actually negative. *D* was false negative, meaning that the actual result was positive, but actually negative. *M* was the error rate.

The article "Account of Deep Learning-Based Ultrasonic Image Feature in the Diagnosis of Severe Sepsis Complicated with Acute Kidney Injury" was retracted in 2023. Reasons: signs of a paper mill; suspected computer-generated content; unreliable results or conclusions; concerns about the data.

Receiver-operating characteristic (ROC) curve was used to represent the diagnostic efficiency of the three algorithms and artificial diagnoses of professional physicians. The area under curve (AUC) of ROC was determined according to ROC. Comparative analyses were conducted.

### 2.5. Statistical Methods

SPSS 24.0 software was used for statistical analyses of data. Data conforming to normal distribution was expressed as mean ± standard deviation (mean ± *s*), *t* test was used to represent measurement data, chi-square (*χ*^2^) test was used to represent count data, and *P* < 0.05 indicated statistical differences.

## 3. Results

### 3.1. Ultrasonic Image Results of Severe Sepsis Complicated with Acute Kidney Injury

Ultrasound image examinations were performed on patients with severe sepsis complicated with acute kidney injury.  Figure 4 showed some patients' ultrasound images. The results showed that many patients had multiple renal injuries which included abnormal renal morphology, renal parenchymal area deformation, renal capsule damage, and diffuse renal enlargements. In severe cases, the kidney was obviously swollen, the morphology and structure of the kidney were seriously changed or even became abnormal, the internal structure of each became incomplete or even disappeared, and the outline was not clear, showing the disorder of light like mass.

### 3.2. Ultrasonic Image Diagnostic Test Results on account of Deep Learning

As shown in Figure 5 below, the accuracy of the ResNet, GoogLeNet, and DenseNet121 algorithms was 95.8%, 95.3%, and 96.1%, respectively; which were significantly higher than the 91.6% of manual diagnosis by specialists (*P* < 0.05). The sensitivity of three algorithms was 92.3%, 91.8%, and 93.4%, respectively, higher than that 84.5% of the manual diagnosis by specialists significantly (*P* < 0.05). In terms of specificity, there was no significant difference among the three algorithms and the manual diagnosis (*P* > 0.05).

The article "Account of Deep Learning-Based Ultrasonic Image Feature in the Diagnosis of Severe Sepsis Complicated with Acute Kidney Injury" was retracted in 2023. Reasons: signs of a paper mill; suspected computer-generated content; unreliable results or conclusions; concerns about the data.

The misjudgment rate of sepsis complicated with acute kidney injury was 5.2%, 6.3%, and 4.9% of the ResNet, GoogLeNet, and DenseNet121 algorithms, respectively. These were all significantly lower than the 14.5% of that by specialists manually, with the difference statistically significant (*P* < 0.05). It could be observed in Figure 6 for details.

### 3.3. ROC Curve and AUC Comparison Results

According to the three algorithms and the specificity and sensitivity of professional doctors' artificial diagnoses, ROC curves were drawn, which were shown in Figure 7.

After determining and comparing AUC of ROC, AUC of professional physicians' diagnoses was 0.896, significantly lower than that of the three algorithms on account of deep learning. The specific results were shown in Figure 8.

### 3.4. The Loss Function Results of the Improved Algorithms

The loss function of DenseNet121 algorithm converged after about 650 times after comparing the training loss function of the three algorithms. However, the training loss of ResNet and GoogLeNet algorithms reached convergence after 700 times. Specific results were shown in Figure 9.

At the same time, training time and the number of parameters of the three algorithms were compared and analyzed; there were no significant differences in training time. However, the number of DenseNet121 and GoogLeNet parameters was significantly lower than that of ResNet algorithm (*P* < 0.05), which were shown in Figure 10.

## 4. Discussions

At present, the incidence and mortality of severe sepsis complicated with acute kidney injury are gradually increasing. Clinically, it is very important for the early diagnosis and treatment of sepsis complicated with acute kidney injury. Delays in early diagnoses and treatments lead to the progression of the disease, worsening its progression, causing irreversible damage, and rapidly leading to death. Therefore, accurate diagnoses and examination are extremely important [26]. 50 patients with severe sepsis complicated with acute kidney injury and 50 healthy volunteers were selected in this study. They all underwent ultrasound scans. Different deep learning convolutional neural network models DenseNet121, GoogLeNet, and ResNet were used for training and diagnoses. Then, diagnostic results were compared with professional image physicians' artificial diagnoses. Results showed that the accuracy and sensitivity of three algorithms on account of deep learning were significantly higher than professional physicians' artificial diagnoses (*P* < 0.05). However, there were no significant differences in specificity between the two groups (*P* > 0.05). At the same time, the error rate of the three algorithm models for severe sepsis complicated with acute kidney injury was significantly lower professional doctors' artificial diagnoses (*P* < 0.05). AUCs of the three algorithms were significantly higher than doctors' diagnosis results (*P* < 0.05). Compared with clinicians' artificial visual diagnoses, deep learning-based convolutional neural network models could identify ultrasonic image features more accurately and had greater value for the clinical diagnoses of severe sepsis complicated with acute kidney injury.

The article "Account of Deep Learning-Based Ultrasonic Image Feature in the Diagnosis of Severe Sepsis Complicated with Acute Kidney Injury" was retracted in 2023. Reasons: signs of a paper mill; suspected computer-generated content; unreliable results or conclusions; concerns about the data.

As a kind of deep neural network, convolutional neural network could transform image data into visual pathological features and obtain information that could not be directly captured by human eyes, which was extremely important in ultrasound clinical diagnoses [27]. In this study, three convolution neural network models DenseNet121, GoogLeNet, and ResNet were used to process and analyze the ultrasound images of patients with severe sepsis complicated with acute kidney injury. The results showed that ResNet and GoogLeNet algorithms converged after 700 times, while DenseNet121 algorithm needed 650 times to converge. There were no significant differences in training time between the three algorithms on account of deep learning (*P* > 0.05). However, the number of parameters of DenseNet121 and GoogLeNet was significantly lower than that of ResNet (*P* < 0.05). In addition, the results showed that the error rate of professional physicians in clinical diagnoses of severe sepsis complicated with acute kidney injury was as high as 15.01%. The error rate of DenseNet121, GoogLeNet, and ResNet was 4.98%, 6.75%, and 5.32%, respectively, which were significantly lower than professional physicians' artificial diagnoses (*P* < 0.05). Le et al. (2021) [36] pointed out after experiments that the accuracy and sensitivity of the diagnosis were higher than that of the doctor as the convolutional neural network was optimized, which is consistent with the results of this study. In conclusion, the value of the three algorithms on account of deep learning in the diagnoses of severe sepsis complicated with acute kidney injury by ultrasonic image features was higher than the artificial judgment of professional physicians, which had great clinical value for the diagnoses and treatments of the disease. However, the diagnoses of any disease require a comprehensive judgment on account of clinical symptoms, signs, professional experience, and image examination. Therefore, comprehensive evaluation should be combined with many factors in the clinical diagnoses of severe sepsis complicated with acute kidney injury.

The article "Account of Deep Learning-Based Ultrasonic Image Feature in the Diagnosis of Severe Sepsis Complicated with Acute Kidney Injury" was retracted in 2023. Reasons: signs of a paper mill; suspected computer-generated content; unreliable results or conclusions; concerns about the data.

## 5. Conclusions

50 patients with severe sepsis complicated with acute kidney injury and 50 healthy volunteers were selected in this study. They all underwent ultrasound scans. Different deep learning convolutional neural network models DenseNet121, GoogLeNet, and ResNet were used for training and diagnoses. Then, the diagnostic results were compared with professional image physicians' artificial diagnoses. The results showed that the accuracy and sensitivity of the three algorithms on account of deep learning were significantly higher than professional image physicians' artificial diagnoses. At the same time, the error rate of the three algorithm models for severe sepsis complicated with acute kidney injury was significantly lower than professional doctors' artificial diagnoses. In addition, among the three algorithms, DenseNet121 was easier to achieve convergence, and the number of parameters of DenseNet121 and GoogLeNet was significantly lower than that of ResNet. In conclusion, the value of the three algorithms on account of deep learning in the diagnoses of severe sepsis complicated with acute kidney injury by ultrasonic image features was higher than professional doctors' artificial diagnoses, which had great clinical value for the diagnoses and treatments of the disease. The shortcomings of this study are that the sample size of the research object is small, and the source is single, which does not have randomness and wide applicability. In the future, multisite, multitype, and large-sample analyses and researches will be considered to provide more practical. In short, the three algorithms under deep learning were more valuable in the diagnosis of severe sepsis complicated with acute kidney injury than the specialists, and they gave important clinical value in the diagnosis and treatment of the disease. This study provided a reference for the imaging diagnosis of sepsis complicated with acute kidney injury.

## Figures and Tables

**Figure 1:** DenseNet121 convolutional neural network model.

**Figure 2:** The inception module of GoogLeNet.

**Figure 3:** ResNet convolutional neural network model.

**Figure 4:** Ultrasonic image results of severe sepsis complicated with acute kidney injury.

**Figure 5:** Comparison of accuracy, specificity, and sensitivity between the three algorithms and professional physicians. Note: ^∗^ represented significant differences: *P* < 0.05.

**Figure 6:** Comparison of the error rates among the three algorithms and professional physicians. Note: ^∗^ represented significant differences: *P* < 0.05.

The article "Account of Deep Learning-Based Ultrasonic Image Feature in the Diagnosis of Severe Sepsis Complicated with Acute Kidney Injury" was retracted in 2023. Reasons: signs of a paper mill; suspected computer-generated content; unreliable results or conclusions; concerns about the data.

**Figure 7:** ROC curve results of the three algorithms and diagnoses by professional physicians.

**Figure 8:** Comparison results of AUCs between the three algorithms and professional doctors' diagnoses. Note: ^∗^ represented significant differences: *P* < 0.05.

**Figure 9:** Loss function of the three algorithm models.

**Figure 10:** Comparison results of training time and parameter number of the three algorithms. Note: ^∗^ represented significant differences: *P* < 0.05.

## Data Availability

The data used to support the findings of this study are available from the corresponding author upon request.
